This article has been retracted.

# Experimental Study on the Effect of Taijiquan on the Physical Function and Mental Health of College Students

**DOI:** 10.1155/2022/7346946

**Published:** 2022-09-21

**Authors:** Meixing Gao

**Affiliations:** College of Physical Education, Shihezi University, Shihezi, 832000 Xinjiang, China

## Abstract

With the continuous development of education and economy, people pay more and more attention to the improvement of comprehensive quality. College students are a special social group. Now they are not only under enormous pressure of study and employment but also pay more attention to physical function and mental health. Maintaining healthy physical fitness is one of the goals pursued by more and more college students. This paper studies the effects of Tai Chi on the physical and mental health of college students. Taijiquan is a physical education class, divided into an experimental group and a control group. The experimental group was trained three times a week, and the control group was trained once a week. Through the evaluation of college students who practice Tai Chi three times a week and college students who practice Tai Chi once a week, the conclusions are: first, there are significant differences in lung capacity, one-minute skipping rope, and sitting forward bending; second, in self-esteem on assessment, significant differences were found in visual perception threshold ability, somatization, and anxiety factors. The final results are as follows: after 8 weeks of Taijiquan practice, the effect of the experimental group and the control group on the spirometry test (*P* > 0.05) and the difference in sitting flexion index between male and female students were statistically significant (*P* < 0.05); Taijiquan was practiced with different frequencies for 8 weeks. After that, the number of skipping ropes did not increase significantly (*P* < 0.05). That is, different frequencies of Taijiquan practice have an impact on the physique of college students. Taijiquan exercise also has a significant impact on the visual perception threshold ability, which can effectively reduce the somatization, paranoia, anxiety, depression, and other psychological states of college students.

## 1. Introduction

With the rapid development of education and social economy in our country, the society has put forward higher and higher requirements for professional ability and comprehensive quality of talents. Modern college students are facing enormous pressure from study and employment competition. Based on the health of students and the strategic position of the state giving priority to education, in the process of promoting economic construction and development, we will develop education and human resources, build a strong country, improve people's livelihood, and realize the great rejuvenation of the Chinese nation: social development. With the continuous development of society, the pace of people's work and life is gradually accelerated, and the pressure in all aspects is gradually increasing; in this case, people have fewer and fewer opportunities to participate in sports activities, which has a negative impact on people's health. Therefore, good physique and health reserves are very important for college students' future employment and even work. However, a large number of research data show that today's college students have insufficient health awareness, insufficient understanding of health knowledge, lack of good and scientific fitness concepts, lack of investment and participation in physical education, and college students' physical fitness has declined significantly. Overweight, obesity, myopia, and other modern civilization the disease gradually increased. The continuous development of society and the high requirements of education on the comprehensive quality of talents have formed a clear contradiction with the decline of college students' physical quality.

Taijiquan is one of the representatives of traditional Chinese national sports. The 24-style Taijiquan proposed by Yang's Taijiquan aims to enhance the fitness of the whole people and improve the quality of life of the whole people. 24-Style Taijiquan generally refers to simplified Taijiquan. It is one of the traditional boxing techniques and belongs to the simple Taijiquan routines implemented after the founding of the People's Republic of China. It has rich connotations and contains the traditional culture and philosophy of the Chinese nation. After long-term promotion and popularization, it has a good mass base. Boxing is not only the essence of Taijiquan but also has three major functions: brain training, qi training, and body training. Therefore, it has a great impact on the human body. At the same time, 24-style Taijiquan has the characteristics of easy learning, small constraints, strong safety, and strong controllability [1]. The measurement of exercise intensity can be adjusted according to the needs of different groups of people. Therefore, it is suitable for promotion and practice in schools to benefit students for life. At present, most colleges and universities have set up Taijiquan elective courses, most of which take 24-style Taijiquan as the main teaching and practice content. According to the characteristics of 24-style Taijiquan being relatively simple and easy to learn, it is widely used in colleges and universities. Tai Chi is becoming more and more popular in China. It integrates various boxing methods of the past dynasties, combines ancient Daoyin and breathing techniques, and absorbs classical philosophy and traditional Chinese medicine theory. In recent years, Tai Chi has become popular among middle-aged and elderly people, but not among young people. At the same time, on the other side of the world, more and more people are discovering that Tai Chi is used for fitness and entertainment and gains new life motivation from it. Practicing Tai Chi is very helpful for Westerners, because it can not only learn some physical and mental skills but also change people's mentality and learn traditional Chinese sports culture. Taijiquan is more and more popular with foreigners, and its influence spreads all over the world. Various styles of Taijiquan have appeared abroad, making Taijiquan culture widely spread around the world. Tai Chi is widely used in Japan, the United States, Canada, the United Kingdom, France, Sweden, Singapore, Malaysia, and other countries as well as Hong Kong, Macao, and Taiwan regions. Tai Chi has spread to more than 140 countries and regions and has gradually become a worldwide health sport. At present, many foreign scholars are also studying the influence of Taijiquan on physical and mental health.

A number of experimental results show that moderate aerobic exercise can effectively improve people's physical and mental health. The fitness function of Tai Chi has been proven and incorporated into modern medicine. At present, the influence of Taijiquan on mental health is mainly concentrated on middle-aged and elderly people and college students. But there are no reports on the effects of Taijiquan on the mental health of middle-aged menopausal women. More research has focused on Tai Chi's effects on the mental health of middle-aged and elderly people. Others conducted mental health checks on 182 middle-aged and elderly people in Beijing. The results show that physical exercise does not completely improve depression in middle-aged and elderly people [2]. They believe that the emotions of middle-aged and elderly people are relatively stable, and it is not easy to change greatly with changes in the environment. However, different studies have different views. Some people use SCL-90 (Symptom Checklist 90 [3]) and POMS (Emotional State Scale) to compare and analyze the influence of Taijiquan before and after practice on the mental health of college students. After 7 months of Taijiquan practice, the patient's mental health has changed, and the scores of each factor are lower than before. Pre-exercise somatization [4], hostility, paranoia, and psychosis were significantly lower than pre-exercise. The factors such as compulsion, interpersonal relationship, depression and anxiety were significantly lower than those before Taijiquan, indicating that Taijiquan has a positive effect on improving the mental health of college students.

This paper studies the influence of Tai Chi on the physical quality and mental health of college students. Taijiquan was the research object, and the subjects were divided into an experimental group and a control group. The experimental group was trained three times a week, and the control group was trained once a week. By evaluating college students who practiced Taijiquan 3 times a week and Taijiquan once a week, the following conclusions were drawn: there were significant differences in lung capacity, 1-minute skipping rope, and sitting forward flexion; in self-assessment, visual perception threshold ability [5], there were significant differences in somatization and anxiety factors. Some scholars have pointed out that “mental health” is a state of good life adaptation. Most mentally healthy people can meet the following conditions: (1) emotional stability, no long-term anxiety, less psychological conflict; (2) willing to work, able to show their talents in work; (3) able to establish harmonious relationships with others, willing to work with others communication with others; (4) have a correct understanding of oneself and an attitude of self-acceptance; and (5) a correct understanding of the living environment can effectively face and solve problems, rather than escape [6]. In the definition of the concept of mental health, it can be said that mental health is actually a long-term sustained psychological state, which is characterized by a good state of mind, emotional stability, and correct interpersonal relationships. We should have a more complete organization and plan to ensure the implementation of health promotion. The goal is to create a healthy campus environment, cultivate students' good health awareness and habits, and a supporting support system.

## 2. The Experimental Research Plan of Taijiquan on the Physical Quality of College students

### 2.1. General Framework of the Research Plan

Taijiquan is one of the most representative sports in traditional Chinese sports, which has the function of fitness and disease prevention. The 24-style Taijiquan routines are arranged according to the principle of easy to difficult. The research on the influence of Taijiquan on the physical health of college students is mainly the research on body function. Most of the research on the influence of Taijiquan on the physical health of college students is on the qualitative description of its fitness effect. The selection of physical fitness testing indicators [7] is not sufficient, and further research and improvement are needed. This research uses the experimental method of Taijiquan training for college students to test and analyze the physical health indicators that can reflect the body shape, physical function, and physical quality of college students, and to study the impact of Taijiquan on physical function [8] and the quality of college students.

### 2.2. Research Objects

As shown in Table 1, 24-style Taijiquan was used to study the physical fitness test indicators of college students. The subjects were divided into experimental and control groups. The experimental group was trained three times a week, and the control group was trained once a week for physical function and mental health. The ratio of male to female in the two experimental groups was 30. The female was 18 years old and the male was 19 years old; the height of the female was 160–165 cm, and the height of the male was 167–172 cm; the weight of the female was 52–55 kg, and the weight of the male was 57–62 kg.

### 2.3. Research Methods

Select and recruit students from the Class of 2019 as volunteers. There are 50 men and 50 women, for a total of 100 candidates. By measuring the physical health indicators before and after 8 weeks of 24-style Taijiquan training, the impact of Taijiquan practice on the physical health test indicators of college students was analyzed. The basic information of the experimental and control groups is shown in Table 1.

The subjects were randomly divided into two groups. The details are as follows: The first group was the control group. Tai Chi training classes are scheduled once a week. The second group is the experimental group, arranged three times a week.

During the training process, the training measurements of the two groups of students were controlled, and each class was 90 minutes long.

### 2.4. Selection of Test Indicators

The measurement of physical function and quality of college students mainly includes physical function and physical quality. Physical function refers to the life activities of the whole human body and its various organs and systems. The development of bodily functions can enhance the strength of the respiratory muscles and increase the range of thoracic movements, thereby improving the respiratory function. (1) The index reflecting the physical function is the lung capacity test; and (2) the index reflecting the physical condition is: sitting forward bending, skipping rope for one minute. Considering the sensitivity of the indicators, the main test indicators in this experiment include lung capacity, and three indicators according to the National Student Physical Health Standard [9] and the College Student Physical Health Standard.

The instruments required for the experiment are as follows: mid-body verticality tester, air volume tester (20084344), stepping tester (20084317), sitting flexion tester (20084315), and skipping rope tester (20107433).

### 2.5. Overview of the Constitution

Physique is the quality of the human body. Physical fitness generally refers to the strength, speed, endurance, sensitivity, flexibility, and other functions of the human body in activities; physical fitness is the external manifestation of a person's physical strength. It is a relatively stable characteristic based on a combination of genetic and acquired human body shape, physiological functions, and psychological factors. There are many factors that affect physical fitness, among which genetics, nutrition, and physical exercise play an important role. A person's physical quality is usually expressed as the body's morphological structure, physiological function, and physical quality.

The developmental level of body shape includes body shape, posture, nutritional status, and body shape; the physiological function level refers to the metabolic level of the body and the working ability of organ systems; the developmental level of physical fitness and athletic ability includes cardiorespiratory endurance, flexibility, muscle strength and endurance, speed, explosiveness, balance, sensitivity, coordination, and reaction time.

### 2.6. Physical Fitness Test Standards for College Students

The “National Student Physical Health Standards” was officially promulgated and implemented in April 2007. It plays an important role in strengthening quality education, promoting college students to master the basic knowledge and scientific methods of physical exercise, improving students' physical health, and promoting development: student sunshine movement. According to the requirements of the National Student Physical Health Standard, college students are required to complete project tests, including height, weight, vital capacity, 1000 m run (male), 800 m run (female), sitting posture, throwing medicine ball, sitting up (female), pull-up (male)), standing long jump, skipping rope, basketball dribble, football dribble, volleyball mat, etc.

In this paper, according to the National Student Physical Health Standard and the College Student Physical Health Standard, the main test indicators of the experiment include lung capacity, sitting forward bending, and 1-minute skipping rope.

## 3. Experimental Research Plan on the Influence of Taijiquan on the Mental Health of College Students

### 3.1. Overview of the Research Plan

With the continuous development of society and the continuous improvement of people's living standards, competition in various industries is becoming increasingly fierce. People are in a state of tension for a long time, and the psychological pressure is also increasing. Especially college students, one of the special groups in society, are far from objective and subjective reality. They cannot fulfill all kinds of wishes. There are many things, many words, and some personal privacy that cannot be told to others very well. For a long time, they could not let go of the pain accumulated in their hearts. As a result, they often feel aggrieved, pessimistic, and world-weary. The study found that college students who do not practice Taijiquan have nowhere to escape due to study and environmental problems, causing trouble. For students who practice Tai Chi, they can not only feel the joy of practicing Tai Chi but also relieve stress. Taijiquan exercises people's internal organs by emphasizing calming the mind, eliminating distracting thoughts, and allowing people to concentrate during exercise. Through reverse abdominal breathing, combining movement, and stillness, the brain relaxes and the central nervous system can self-repair and regulate itself. Taijiquan exercise can soothe the mind and, at the same time, make the human body under a suitable exercise load. Good stimulation is beneficial. Based on the secretion of male hormones, the human body can produce a happy and peaceful feeling and eliminate unpleasant emotions. Confidence is a good standard behavior and also serves as a platform for making friends. Good interpersonal relationships are one of the important indicators to measure mental health, and it is also an important condition for mental health to remain stable. Harmonious communication with friends is conducive to improving people's communication skills and social adaptability [10]. It can effectively reduce the sense of loneliness and realize the happiness of mutual help in practice. It is also the need for social interaction and good interpersonal relationships, which is more conducive to diluting the troubles in life and work, and eliminating stress and loneliness. Establish the desire for life and the unremitting pursuit of beautiful things, and be full of hope and future for everything. This research uses the experimental method of the influence of Taijiquan training on the mental health of college students, to test and analyze the psychological health level of college students, so as to reflect the psychological quality of college students, and to study the influence of Taijiquan on the psychological health level of college students.

### 3.2. Research Objects

In this paper, 24-style Taijiquan [11] is used to study the mental health level of college students. Taijiquan is the object of physical education class, divided into experimental group and control group. The experimental group was trained 3 times a week, and the control group was trained once a week to affect the level.

### 3.3. SCL-50 Questionnaire

Select and recruit students from the Class of 2019 as volunteers. There are 50 men and 50 women, for a total of 100 candidates. By measuring the physical health indicators before and after 8 weeks of 24-style Taijiquan training, the influence of Taijiquan practice on the mental health of college students was analyzed. The level of difference in visual perception thresholds was tested, and mental health was assessed according to the scoring criteria.

The SCL-50 consists of 5 factors and 50 questions. Each factor reflects some aspect of a patient's symptoms and pain. The distributional characteristics of symptoms can be understood by factor scores. Factor 1: somatization (1, 4, 12, 27, 40); factor 2: interpersonal sensitivity (6, 21, 34, 36, 37); Factor 3: depression (5, 14, 15, 20, 22); factor 4: anxiety (2, 17, 23, 33, 39); factor 5: paranoia (8, 18, 43, 68, 76); evaluation method: divided into five levels.

Score (0 to 4), 0 = none, 1 = mild, 2 = moderate, 3 = very severe, and 4 = severe.

### 3.4. Subject Grouping

The subjects were randomly divided into two groups. The details are as follows:

(1) The first group was the control group. Tai Chi training classes are scheduled once a week.

(2) The second group is the experimental group, arranged 3 times a week.

During the training process, the training measurements of the two groups of students were controlled, and each class was 90 minutes.

The visual perception threshold of college students was measured by the digital spot flicker meter of Peking University Instrument Factory.

### 3.5. Selection of Test Indicators

Long-term practice of Taijiquan can continuously improve the system function of various organs of the body and improve the metabolism of the human body. Filling the body with qi and blood and breathing deeply, thinly and evenly is a powerful guarantee for the health of the body. The research on the influence of Taijiquan on the mental health of college students mainly includes testing the visual perception threshold, somatization and anxiety factors, and evaluating the mental health level according to the scoring standard.

Visual perception threshold refers to the minimum brightness contrast that the observer can identify the target from the background, which is related to factors such as the angular width of the target, the brightness of the background, and the probability of expected discovery. The test procedure and method: Under normal circumstances, student volunteers sit in front of the digital light point flicker and turn the flicker meter to the red indicator light. The background light is 1 : 14, the light intensity is 1 : 7, and the light-to-black ratio is 1 : 1. The subjects put their eyes close to the observation port of the flicker meter, and while observing the red indicator light, they turned their fingers to the FM key to observe the red indicator light flashing. Repeatedly adjust between blinking and nonflashing until the red indicator light is not blinking. The higher the average, the better the visual perception. Measure five times. The testers carefully recorded the experimental results. Volunteers were replaced and the experiment continued. Recording: The tester records the test data and calculates the average value. Do not tell the student volunteer test results during the experiment. Change volunteers and repeat the experiment to calculate the average result.

Somatization refers to a person who originally has emotional problems or psychological disorders, but does not manifest as psychological symptoms, but is converted into various physical symptoms. The steps and methods: Under normal circumstances, the student volunteers stand in front of the reaction time exercise time meter, and the tester will reset the number of the control panel to 0. Subjects stared at the indicator buttons, including a red reaction time button and 10 exercise time buttons. Student volunteers press digital buttons on the console at random. After listening to the instructions, the student volunteers pressed the red instruction button. When the red light is on, quickly press the next light button. Two tests and five measurements. The testers carefully recorded the experimental results. Student volunteers were replaced and the experiment continued. Recording: The tester records the test data and calculates the average value. Do not tell the student volunteer test results during the experiment. Change subjects and repeat the experiment to calculate the average result.

### 3.6. Visual Perception Threshold

Minimal detectable stimulus. That is, light, sound, pressure, or other physical quantities, all of which can produce the smallest perceptions, and the smallest stimuli can also produce perceptions. Sensitivity is the ability of people to perceive stimuli. The basic index of detection sensitivity is called the sensory threshold, which is a critical value; the sensory threshold is the critical value of the stimulus intensity required for a person to feel the presence or change of a certain stimulus; the sensory threshold is inversely proportional to the sensitivity.

### 3.7. Somatization

The so-called somatization is such a phenomenon: patients consciously have very serious physical symptoms, such as headache, fatigue, insomnia, physical discomfort, decreased work efficiency, etc., but no obvious lesions are found in the corresponding physical examination or pathological examination. Changes in clinical examination did not explain the severity of the patient's subjective symptoms. The underlying reason for this somatization is that psychological problems have not been solved for a long time.

Everyone expresses their existence and difficulties in different forms in life, and disease is also a way of expression. We know there are physical and mental illnesses. Physiological diseases [12] can cause psychological reactions, and mental diseases can also cause physiological reactions. These two factors influence each other. Second, there are some physical symptoms without organic diseases, mainly caused by psychological and emotional problems, or psychological and emotional problems manifested by physical symptoms, the so-called somatization problems. The term somatic was coined at the beginning of this century. At the time, it referred to the hypothetical process of physical impairment caused by “deeply rooted” neuroses. Later, Ross [13] described somatization as a mental discomfort manifested through somatic symptoms, mainly caused by sociocultural background, that is, social interpersonal relationships. It is a means of expressing and dealing with social and personal issues. Also known as the tendency to experience and express physical discomfort and symptoms under psychological stress, unsubstantiated by pathological findings. It is also the evolutionary process of “biology, psychology, and society.” Through this process, somatic symptoms are used to express and explain various problems between individuals, and the experience becomes a somatic symptom. In other words, it talks about physical symptoms and expresses social and psychological problems.

### 3.8. Anxiety and Depression

Anxiety is a common emotional experience of college students. Anxiety is an irritable emotion caused by excessive worry about the safety of relatives or one's own life, future, and destiny, etc. It contains anxiety, worry, worry, tension, panic, anxiety, and other ingredients. It is a neuropsychological response caused by an adverse stimulus or an impending event that may have adverse consequences for the environment. Worrying too much can turn into anxiety [14], and excessive anxiety can turn into extreme tension and tension. This inexplicable anxiety is a psychological disorder if you are constantly feeling scared and uneasy, and you cannot tell why. Depression is one of the most common mental illnesses now, with continuous and long-term low mood as the main clinical feature, and is the most important type of mental illness in modern people. Depression is an emotional experience of excessive sadness. There are obvious psychological factors in college students' depression, which are related to problems and setbacks in personal study, communication, and life. Personality defects such as inferiority complex, loneliness, pessimism, indifference, overthinking, heavy dependence, irritability, and emotional fragility are the internal basis of the disease.

## 4. Results and Discussion

### 4.1. The Influence of Taijiquan on the Physical Function and Quality of College Students

After 8 weeks of Taijiquan exercise at different frequencies, the results of various physical fitness indicators before and after exercise of the students in the experimental group and the control group are shown in Figure 1.

As shown in Figure 1, after 8 weeks of Taijiquan practice, the physical function of the experimental and control groups was compared, and the lung capacity index of male and female students was *P* ≈ 0.05, and the sitting forward flexion index was *P* ≈ 0.05. In the 1-minute rope skipping index, there was no significant difference between the experimental and control groups, *P* ≈ 0.05. Among them, there was a difference of 0.04 in the vital capacity index and sitting body flexion index between the male and female students in the experimental and control groups.

### 4.2. The Influence of Taijiquan on the Mental Health of College Students

As shown in Figure 2, the SCL-50 self-assessment test was performed on 100 subjects, and the self-assessment factors were used to conduct self-assessment on the college students who practiced Taijiquan once a week and practiced Taijiquan three times a week. The influence of Taijiquan on the visual perception threshold of college students with different practice frequencies is very obvious, the experimental group *t* = 3.4, meanvalue = 37.63, *P* > 0.05 and the control group *t* = 1.55, meanvalue = 26.45, *P* < 0.05.

### 4.3. SCL-50 Test Form for College Students to Practice Taijiquan at Different Frequencies for One Week

As shown in Figure 3, comparing the factors of SCI-90 scale, menopausal women practicing Taijiquan, not practicing Taijiquan, and college students practicing Taijiquan's mental health status, each factor index is better than the frequency of low-frequency training. Among them, somatization = 4.61, *P* = 0.03, *P* < 0.05; anxiety *x*^2^ = 4.07, *P* = 0.042, *P* < 0.05; depression *x*^2^ = 12.3, *P* = 0.063, *P* > 0.05; somatization and anxiety are different, and depression is significantly different.

The results show that Taijiquan has a positive effect on promoting the mental health and physical health of college students. Through different frequencies of Tai Chi exercise, the psychological health level of the experimental group was significantly better than that of the control group. The influence of Taijiquan on the psychology of college students mainly comes from the frequency of Taijiquan practice. When practicing Tai Chi, the movements should be slow, gentle, and continuous, and the whole body should be relaxed. We can experience every action detail, suggesting that mental activity is based on the central nervous system of the brain, which is beneficial to the mental health of college students. This paper further analyzes the differences in mental health factors of college students who practice Taijiquan once a week and practice Taijiquan three times a week.

### 4.4. Comparison of Somatization Factors among College Students

As shown in Figure 4, the somatization factor is one of the important components of mental health and is one of the important manifestations of physical function. Tai Chi is a slow, uniform aerobic exercise. In practice, abdominal breathing requires “the roof of the tongue, the palate, and the qi sinking into the dantian.” As the diaphragm and abdominal muscles continue to contract and relax, abdominal pressure also changes. Intra-abdominal pressure increases, and venous blood continues to flow back into the right atrium. Instead, when the pressure drops, the blood is pumped into the abdominal cavity. In addition, when practicing Tai Chi, you should pay attention to concentration, relax your mind, move slowly, combine inside and outside, coordinate up and down, and breathe slowly and evenly. This can eliminate the anxiety of students due to stress, reduce the tension of the central nervous system, and cause the blood vessels in the body to relax, promote blood circulation, lower blood pressure, and reduce the burden on the heart. It can also effectively improve the working ability of the cardiovascular and cerebrovascular system so that the blood supply of the heart arteries is sufficient.

## 5. Conclusion

Due to the limitation of objective factors such as course time and objects, it is difficult to monitor students' extracurricular activities. This is the problem of this study, which affects the results of the study to a certain extent. Different frequencies of Taijiquan exercise have different effects on the body shape of college students. Taijiquan exercise once a week has no effect on the body shape of college students, while Taijiquan three times a week has a good effect on the physical function quality of college students, which is worthy of in-depth research and analysis. After 8 weeks of Taijiquan practice for college students, the experimental group and the control group were tested. In terms of physical function, boys and girls had significant effects on the Spirometric Index and Sitting Flexion Index. There was no significant difference between the experimental group and the control group in terms of skipping rope per minute. There were significant differences in visual perception thresholds, anxiety, and somatization. Visual perception thresholds are the basis of perception. External stimuli are perceived by the optic nerve and transmitted to the brain for processing, so as to correctly judge the direction, distance, and placement of the action. The stimulation of the motor receptors acts on the muscles, causing the muscles to contract, prompting the limbs to perform each movement correctly. This requires every functional index to function properly. Taijiquan exercise can effectively exercise the muscles of the whole body, experience the joy of exercise, exercise consciousness under guidance, and eliminate external interference. Focus on the practice, focus on the movement, carefully observe the characteristics of each action, concentrate fully, exercise the body, so as to forget the troubles and relieve the pressure of study. Through the appropriate amount of Taijiquan practice, the problem of unresponsiveness can be effectively alleviated, thereby improving physical exercise ability and self-confidence. The high-frequency practice of Tai Chi has a significant effect on the ability to threshold visual perception. The high-frequency exercise of Taijiquan not only trains the physique of college students but also realizes the integration of body and mind in the practice. Therefore, it can effectively alleviate mental states such as somatization, paranoia, anxiety, depression, etc., and effectively relieve students' physiological function, perception, psychological sensitivity, pessimism, tension, and other phenomena. The development of college students' physical function and mental health has important theoretical and practical significance.

## Figures and Tables

**Figure 1:** The effect of Taijiquan on the physical health index of college students.

**Figure 2:** Visual perception threshold of Tai Chi.

**Figure 3:** College students SCL-90 practicing Tai Chi once a week and 3 times a week.

**Figure 4:** Comparison of somatization factors of college students.

**Table 1:** Basic information table of experimental subjects.

Test group	Gender	Number of people	Age	Height, cm	Weight, kg
Experience group	Female	30	18	160 ± 5	52 ± 3
	Male	30	19	167 ± 5	57 ± 3
Control group	Female	30	18	160 ± 5	52 ± 3
	Male	30	19	167 ± 5	57 ± 3

## Data Availability

The data that support the findings of this study are available from the corresponding author upon reasonable request.
